The article "Determination of the Influence of Strut Connector on Stent Deployment" was published in 2022. Journal: Appl Bionics Biomech.

# Determination of the Influence of Strut Connector on Stent Deployment

**DOI:** 10.1155/2022/7232809

**Published:** 2022-06-28

**Authors:** V. Hashim, S. L. Resmi, P. N. Dileep

**Affiliations:** Department of Mechanical Engineering, TKM College of Engineering, Kerala, India

## Abstract

Coronary artery stents are tubular structures employed together with angioplasty. Stented angioplasty is a clinical procedure widely applied in the treatment of atherosclerosis to reopen the blocked artery. It is a simple and fast curing minimally invasive clinical procedure. However, it is essential to understand the expansion characteristics of a stent before implantation since the stent geometry, inflating pressure, etc., influence the performance of stents. Finite element analysis and in vitro experiments are simultaneously employed before clinical testing to predict the characteristics during deployment. In this paper, the expansion and deployment characteristics of Meril Osum 2.75 × 24 coronary stent and Envision 3.5 × 28 stent were investigated to study the influence of strut connector on the expansion behaviour of the stent by experimental and computational methods. The current study analyzes the real-time deployment characteristics such as rate of expansion, stress on stent, recoil, dog boning, and foreshortening. The stent expansion characteristics obtained from experiments and simulations were found matching and observed that strut connector has a significant effect on stent expansion. Further, the curved connector of small radius of curvature shows better performance with high patency rate.

## 1. Introduction

The most numerous health problem in the present scenario is cardiovascular disease. Angioplasty with stent implantation is a popular treatment for atherosclerosis. The precrimped stent is located at the blocked lesion, and it is expanded using a balloon in this treatment. The plastically deformed stent compresses the plaque which acts as a permanent scaffold to reinstate the blood flow to the heart. The latest developments in stent technology increased its acceptance because of its flexibility and deliverability, and hence, it is possible to deploy even in the complex coronary lesions. Also, emergence of drug-eluting stents (DES) reduced the restenosis rate compared to bare metal stent (BMS) [1]. However, in-stent restenosis (reblocking the stented artery due to thrombosis or calcification) still remains as major challenge in 10-20% of the stented artery. The study found that the geometric design is the major differentiating factor between the available stents which greatly influences the expansion characteristics [2]. In the case of the slotted tube design, length of the slot, slot width, number of slots per circumference, etc. were the significant geometrical parameters [3], whereas strut thickness, crown radius, strut width, etc. were the key parameters for ring and connector type design [4]. Another study by Imani et al. proved that the ring type design with circumferential rings and connector is more efficient in terms of flexibility and radial expansion than slotted tube stent. The strut connectors of different shapes like straight, U, V, and S are available, and S-shaped connector shows better flexibility, maximum expansion, minimum stress, and foreshortening [5–7]. The majority of the studies in this area were based on finite element methods which compare different stent models to evaluate their performance. Some of them were free stent expansion and others within a diseased artery. A typical FE analysis of stent deployment consists of several important preprocessing stages such as generation of FE model, meshing, assigning the material property, and defining the boundary and loading conditions. Finite element analysis is an effective tool to study the expansion behavior of artery stents. It gives accurate information on stent expansion, recoil, dog-boning, foreshortening, and residual stresses. Moreover, this method is implemented effectively to simulate the stent deployment in a diseased artery and conduct parametric study on stent geometry. The analysis on stented artery evaluates the influence of stent design on in-stent restenosis effectively and the output data can be used to optimize the stent geometry accordingly [8, 9]. It was observed that the percentage of dog-boning varies with the length of the balloon and its characteristics. The overexpansion may increase dog boning effect, and the underexpansion will affect the scaffolding action of the stent [10, 11]. The inflating pressure of the balloon also affects the expansion characteristic. Due to its high risk and cost, the experimental and clinical investigation on stent analysis was comparatively rare. Therefore, the computational investigation is predominant in the published work. The effect of connector geometry on the expansion behavior of stents had been systematically explained in this paper both by experimental and computational methods. Finally, it finds the optimum shape of the connector for the given model.

The article "Determination of the Influence of Strut Connector on Stent Deployment" was published in 2022. Journal: Appl Bionics Biomech.

## 2. Materials and Methods

Two types of stents Meril Osum 2.75 × 24 and Envision 3.5 × 28 were used in the proposed experiment. Osum and Envision are widely used stents available in Indian market, and both of the stents are of balloon-expandable with good structural integrity and flexibility. The major difference between these two stent designs is the shape of the connector. Meril Osum has an S-shaped connector whereas Envision has a straight connector. The images of original Osum stent and Envision stent in crimped form are shown in Figures 1 and 2 respectively. The characteristics of both the stents are demonstrated in Table 1.

### 2.1. Experimental Method

The experiment on the expansion characteristic of the coronary stent was conducted at Sree Chitra Tirunal Institute of Medical Sciences and Technology, Trivandrum using an automated instrumentation system as shown in Figure 3. The system is capable of measuring the transient radial displacement with respect to inflation pressure in a controlled environment. It consists of a standard pressure controller (GDS Instruments, UK), a noncontact type optical micrometer (LS 7030 M, M/s. Keyence, Japan), and a fixture for holding the stent and delivery system as shown in Figure 4. The input and output data during the process are recorded and saved in the computer using virtual instrumentation LabVIEW software. Stent together with the delivery system was connected to the pressure controller and the distilled water from the pressure controller of the balloon, and the stent was expanded. Inflating pressure of 912 kPa was set in the pressure controller with a slope of 100 ms/kPa so that it takes 80 s to expand the balloon, and it is held for 24 s (holding time); then, the balloon was deflated to 0 kPa with a slope of 100 ms/kPa.

The optical micrometer measures the outer diameter of the middle of the stent during the timed expansion with an accuracy of +/-0.002 mm, and the data was scanned by the PC application at a rate of 30 samples per second. Both pressure and displacement were measured and recorded using an automated instrumentation system. The geometry of the stent is measured with an optical microscope as shown in Figure 5 both before and after expansion. The geometry of the stent distal end, strut thickness, etc., were measured, and the expansion characteristics like foreshortening, dog-boning, and recoil of the stent were calculated from this geometry. Radial recoil (RR), foreshortening (FS), and dog-boning (DB) are the expansion features of the stent generally taken into consideration in most of the stents. Where RR is the amount of radial shrinkage of the stent during the pressure release due to elastic recoil, FS is the amount of axial reduction in the length after expansion, and DB is the enlargement of diameter on both open ends of the expanded stent with respect to the diameter of the middle section. All three expansion characteristics can be computed using the equations given below:

(1) $$\begin{array}{c} \text{Radial Recoil of stent }\left(\text{RR}\right)=\frac{\left(R_{1\text{central}}–R_{2\text{central}}\right)}{R_{1\text{central}}}, \end{array}$$

(2) $$\begin{array}{c} \text{Foreshortening}=\frac{\left(L_{1}–L_{2}\right)}{L_{1}}, \end{array}$$

(3) $$\begin{array}{c} \text{Dogboning}=\frac{\left(R_{2\text{distal}}–R_{2\text{central}}\right)}{R_{2\text{distal}}}, \end{array}$$

where *L*_1_ and *L*_2_ are the length of the stent before and after expansion, respectively. *R*_2distal_ and *R*_2central_ are the radii of the stent at the end and middle after expansion. *R*_1central_ is the radius of middle of the stent before deflation.

The article "Determination of the Influence of Strut Connector on Stent Deployment" was published in 2022. Journal: Appl Bionics Biomech.

### 2.2. Finite Element Method

A unit cell of Osum stent model with two rings and a connector was created in SOLIDWORKS modelling software. The unit cell model represents the same behavior of full stent model that was confirmed from the trial analysis and from literature [9]. A preliminary analysis was conducted to study the mesh sensitivity by varying the mesh element size from 0.055 mm to 0.030 mm. The nodal stress and displacement were compared for different mesh sizes. It was found that a global mesh size of 0.035 mm and 0.030 mm gives consistent result for stent with no significant changes in the responses, and hence, a mesh size of 0.035 mm was fixed for stent. Similarly, a mesh size of 0.05 mm was found compatible for the balloon, and a fine mesh of 0.015 mm was opted for the crown part of the strut where the deformation was predominant during expansion. The finite element meshed model of the unit cell and balloon assembly of the Osum stent is given in Figure 5. The meshing of the stent was done with 8-node hexahedral brick elements (C3D8R) with a total number of 4914 nodes and 2410 elements.

FE analysis on the expansion of the model was performed in Abaqus CAE 6.14 with loading and boundary conditions similar to the in vitro experiment. A nonlinear static analysis was implemented for stent balloon assembly with a surface to surface contact and of frictional coefficient of 0.25. The analysis was performed in two steps such that the balloon was inflated with a ramp-up load of 912 kPa during first step and deflated with a ramp down in the second step by releasing the balloon pressure to atmosphere. Both steps were performed in equal time interval of 0.8 s without considering holding time. Since the simulation involves material, geometry, and contact nonlinearity, the computation time was quite large; hence, a quarter of the circumference was considered for the simulation. Symmetric boundary conditions were imposed on the stent to enable radial expansion such that all the nodes perpendicular to the plane are arrested along the plane of symmetry as shown in Figure 6. However, both ends of the stent were free from any constraints to account axial displacement. Hence, the foreshortening behavior of the stent was computed. Three different models with different connector curvatures for connector were analyzed for identifying the effect of strut connector on its expansion features.

The article "Determination of the Influence of Strut Connector on Stent Deployment" was published in 2022. Journal: Appl Bionics Biomech.

An elastoplastic material was assumed for the stent to approximately represent the behavior of cobalt-chromium (L-605), and its material properties were chosen as Density = 9.1*e*^−6^ kg/mm^3^, Young′s modulus = 243 GPa, and Poisson′s ratio = 0.30 (Pochrzast et al., 2009). Hyperelastic polyurethane balloon was selected for the balloon, and its deformation behavior was examined under the hyperelastic Mooney-Rivlin strain energy function: *W* = C_10_(I_1_ − 3) + C_01_(I_2_ − 3) + (J − 1)^2^/D_1_, where *I*_1_ and *I*_2_ are the first and second stretch invariants; *J* is the volumetric stretch (or third stretch invariant); *C*_10_, *C*_01_, and *D*_1_ are model parameters with values given in Table 2 (Karimi et al. 2014).

## 3. Results and Discussions

During the inflation stage of the in vitro experiment, the crimped stent starts opening at the ends and propagates towards the middle of the stent axially. The expansion was observed rapid at the beginning and turns to a steady increment with pressure. In the case of Osum 2.75 × 24, a maximum expansion of 2.963 mm was reached at the end of inflation pressure of 900 kPa and the diameter reduced to 2.903 mm at the end of deflation due to elastic recoil. Similarly, a highest diameter of 3.469 mm was obtained for Envision 3.5 × 28 at 800 kPa and reduced to 3.239 mm at the end of deflation. The image of the expanded Osum stent and Envision stent are shown in Figures 7 and 8, respectively.

The shape of the strut has been transformed to trapezoidal on both stents during expansion. The struts moved apart, and the crown was found stretched with an increase in the crown radius. The deformed shape of the struts of Osum and Envision stents are given in Figures 9 and 10, respectively. The geometry of the expanded stent was measured using Leica digital microscope, and the expansion characteristics such as radial recoil, foreshortening, and dog-boning were computed from the Equations (1)–(3), respectively.

Even though the expansion processes were same for both Osum and Envision stents, some differences were noticed in the expansion behavior. This is mainly due to the changes in the stent geometry and the crimping ratio. The rapid expansion at the beginning was due to uncrimping of stent, and then, it undergoes elastic deformation and finally plastic deformation. This is clearly illustrated in the graph shown in Figure 11 for both the stents.

The article "Determination of the Influence of Strut Connector on Stent Deployment" was published in 2022. Journal: Appl Bionics Biomech.

For both the samples, a small percentage of elastic recoil was noted during deflation. The expanded diameter of Envision stent is larger than Osum stent since its initial diameter was larger. The radial recoil of Osum stent was only one-third of Envision stent, which is purely due to geometric effect. Compared to straight connector, the curved connector can promote expansion by stretching the curve by which the recoil and foreshortening is get reduced [6]. A significant difference in foreshortening and dog-boning was also noticed between Osum and Envision stents. Generally, foreshortening increases with expansion rate, whereas the rate of dog-boning mainly varies with the characteristics of balloon and balloon over length. Further, the design of the end strut of the stent influences the dog-boning. In this case, foreshortening and dog-boning of Envision stent show three times larger than Osum stent as observed in Qiao et al. (2014). The expansion characteristics observed from the experimental analysis of both the stents are detailed in Table 3.

The FE analysis was performed in three unit cell stent models A, B, and C. The geometry of Model A exactly same as original Osum stent, and the design of the other two models were similar to Osum stent except the shape of the connector. Model A is of curved connector with a radius of curvature 0.09 mm (“S” type connector), Model B of curved connector with larger radius of 0.12 mm, and Model C with a straight connector. The stress and strain contour of expanded Model A before balloon deflation is given in Figures 12(a) and 12(b), respectively. Similarly the stress and strain contour of the same model after deflation is given in Figures 13(a) and 13(b), respectively. As Model A is very similar to Osum stent, its expansion features shows good correspondences with the experiment. Maximum displacement of 0.731 mm and stress of 677 MPa were obtained at the end of inflation pressure, and it was reduced to 0.645 mm and 461 MPa, respectively, after balloon deflation. The final expanded diameter from computation is 2.960 mm which is very close to the experimental value of 2.961 mm and the FEM was validated.

Figure 14 shows temporal variation of stress and displacement for unit cell model A, and the same behavior was seen in other models also. The maximum displacement was obtained along the radial direction, and a small foreshortening was observed along the axial direction. Curve *U* represent the displacement along the radial direction, *Ux* and *Uy* are the displacement along *X* and *Y* directions, and *Uz* represents the displacement along axial direction which gives foreshortening of stent directly.

The article "Determination of the Influence of Strut Connector on Stent Deployment" was published in 2022. Journal: Appl Bionics Biomech.

Figures 15(a) and 15(b) demonstrate the stress and strain distribution on Model B with curved connector of larger radius. Similarly, Figures 16(a) and 16(b) demonstrate that of the Model C with straight connector. Maximum expansion with minimum stress concentration and recoil was found in the ‘S' curved model. Due to stretching the radius of curvature of the connector increases during expansion until it touches the crown part of the strut. A slight increase in foreshortening and dog-boning was observed in Model A which might be due to the larger expansion rate of the model. Both dog-boning and foreshortening are directly linked with the expansion, and it increases with expansion in normal condition. A better expansion characteristic of Model A is a direct implication of its clinical patency rate. The stent with similar design of Model A will have high patency rate with minimum chance of in-stent restenosis due to less induced stress on artery and low percentage of recoil and foreshortening. Similar observation was found by Qiao et al. (2014).

The poor performance of Model B may be due to the rigidity of the connector which prevents the movement of the strut. Moreover, the orientation of the connector is almost perpendicular to the stent axis which always opposes the radial expansion. The expansion characteristics of the three models were computed from the output using equations (1)–(3). Maximum stress on stent, displacement, recoil, foreshortening, and dog-boning were compared as shown in Table 4.

Further investigation was performed to determine the optimum curvature of the connector using FE analysis. Eight unit cell models with various curvatures were modelled, and the major expansion characteristics: maximum stress, maximum displacement, and recoil, were computed for performance evaluation. Foreshortening and dog-boning were not considered since influence of both on expansion feature was found less significant. Using Minitab statistical software, a correlation function was derived for stress and recoil. The optimum value of the connector curvature for a minimum value of stent recoil and stress was found from this equation. The optimum value of connector curvature obtained was 0.108 mm for the model used for the study, and the optimum curvature may change with the changes in shape and geometry.

## 4. Conclusions

The study compares the expansion characteristics of two different stent designs by experimental methods and found that the stent with S-curved connector gives better expansion characteristics. The results obtained from experiment found good agreement with computational results. The expansion behavior of stent models obtained from FEM also gives better performance for unit cell model with S-shaped connector. It performed well with maximum expansion, minimum stress, low recoil, and less foreshortening. Further, the study computed the optimum value of the connector curvature for the stent considered for the study. The study concludes that shape of the strut connector has a great impact on its expansion behavior. The curved connector can stretch and can promote the expansion process. The effectiveness of the connector depends on the radius of curvature and its orientation. The connector with minimum radius of curvature and orientation along the axis is always better for easy deployment and postdeployment performance.

The article "Determination of the Influence of Strut Connector on Stent Deployment" was published in 2022. Journal: Appl Bionics Biomech.

## Figures and Tables

**Figure 1:** Osum stent (crimped).

**Figure 2:** Envision stent, 3.5 × 28 (crimped).

**Figure 3:** Schematic sketch of the experiment setup (courtesy: Sujesh et al. 2013).

**Figure 4:** Experimental setup.

**Figure 5:** Meshed model of unit cell-balloon assembly.

**Figure 6:** FE model with loading and boundary condition.

**Figure 7:** Expanded Osum stent.

**Figure 8:** Envision 3.5 × 28 stent after expansion.

**Figure 9:** Strut of Osum 2.75 × 24 after expansion.

**Figure 10:** Strut of Envision 3.5 × 28 after expansion.

**Figure 11:** Stent expansion with pressure.

**Figure 12:** (a) Model A: stress distribution before deflation. (b) Model A: strain distribution before deflation.

**Figure 13:** (a) Model A: stress distribution after deflation. (b) Model A: strain distribution after deflation.

**Figure 14:** Variation of displacement and stress with time.

**Figure 15:** (a) Stress distribution on stent with slight curved connector. (b) Strain distribution on stent with slight curved connector.

**Figure 16:** (a) Stress distribution on stent with straight connector. (b) Strain distribution on stent with straight connector.

**Table 1:** Stent characteristics.

Characteristics	Osum 2.75 × 24	Envision 3.5 × 28
Outer diameter	1.03 mm	1.08 mm
Strut thickness	85 *μ*m	73 *μ*m
Length	24 mm	26 mm
No. of rings	18	21
Strut width	80 *μ*m	Variable (80 *μ*m-120 *μ*m)
Strut connector	‘S' type	Straight
Material	L605 cobalt chromium	L605 cobalt chromium

**Table 2:** Material properties of balloon.

Material	Density (kg/mm^3^)	*C*_10_	*C*_01_	*D*_1_
Polyurethane	1.07*e*^−6^	1.03	3.69	0

**Table 3:** Expansion characteristics of Osum and Envision stents from experiment.

Stent	Diameter of stent (mm)			Stent length before expansion (mm)	Stent length after expansion (mm)	Radial recoil (%)	Fore-shortening (%)	Dog-boning (%)
	Before deflation	After deflation	At distal end					
Osum 2.75 × 24	2.963	2.903	2.961	24	23.416	2.02	2.43	1.96
Envision 3.5 × 28	3.469	3.239	3.459	28	26.229	6.63	7.62	6.32

The article "Determination of the Influence of Strut Connector on Stent Deployment" was published in 2022. Journal: Appl Bionics Biomech.

**Table 4:** Expansion characteristics of stent models with different strut connectors from simulation.

Stent model	Maximum stress after deflation (MPa)	Maximum radial displacement (mm)		Radial displacement at the middle (mm)	Axial displacement due to expansion (mm)	Radial recoil (%)	Foreshortening (%)	Dog-boning (%)
		Before deflation	After deflation					
Model A	461	0.731	0.645	0.617	-0.049	5.49	1.56	1.89
Model B	484	0.678	0.569	0.539	-0.057	7.20	1.81	2.13
Model C	484	0.685	0.581	0.558	-0.044	6.84	1.40	1.63

## Data Availability

All data related with experiment and simulation are available and can be produced on demand.
